# Breast MRI Tumor Automatic Segmentation and Triple-Negative Breast Cancer Discrimination Algorithm Based on Deep Learning

**DOI:** 10.1155/2022/2541358

**Published:** 2022-08-31

**Authors:** Ying-Ying Guo, Yin-Hui Huang, Yi Wang, Jing Huang, Qing-Quan Lai, Yuan-Zhe Li

**Affiliations:** ^1^Department of CT/MRI, The Second Affiliated Hospital of Fujian Medical University, Quanzhou 362000, China; ^2^Department of Neurology, Jinjiang Municipal Hospital, Quanzhou 362000, China

## Abstract

**Background:**

Breast cancer is a kind of cancer that starts in the epithelial tissue of the breast. Breast cancer has been on the rise in recent years, with a younger generation developing the disease. Magnetic resonance imaging (MRI) plays an important role in breast tumor detection and treatment planning in today's clinical practice. As manual segmentation grows more time-consuming and the observed topic becomes more diversified, automated segmentation becomes more appealing. *Methodology*. For MRI breast tumor segmentation, we propose a CNN-SVM network. The labels from the trained convolutional neural network are output using a support vector machine in this technique. During the testing phase, the convolutional neural network's labeled output, as well as the test grayscale picture, is passed to the SVM classifier for accurate segmentation.

**Results:**

We tested on the collected breast tumor dataset and found that our proposed combined CNN-SVM network achieved 0.93, 0.95, and 0.92 on DSC coefficient, PPV, and sensitivity index, respectively. We also compare with the segmentation frameworks of other papers, and the comparison results prove that our CNN-SVM network performs better and can accurately segment breast tumors.

**Conclusion:**

Our proposed CNN-SVM combined network achieves good segmentation results on the breast tumor dataset. The method can adapt to the differences in breast tumors and segment breast tumors accurately and efficiently. It is of great significance for identifying triple-negative breast cancer in the future.

## 1. Introduction

Among the new cases of female malignant tumors, breast cancer accounts for as high as 29%, and the mortality rate ranks second in cancer mortality [1]. Breast cancer is a systemic disease with local manifestations. There is currently no effective preventive method for breast cancer. Early detection and early treatment are the only effective means to improve postoperative survival [2]. Breast cancer mainly relies on microvascular oxygen supply. However, in the early diagnosis, due to the early manifestations of malignant lesions and the enhancement of benign lesions, the specificity of the disease is poor [3–5]. In recent years, molecular typing of breast cancer has become a research hotspot because different molecular types of breast cancer have significant differences in disease expression, response to treatment, prognosis, and survival outcomes. Triple-negative breast cancer is defined as breast cancer that is immunohistochemically negative for estrogen receptor (ER), progesterone receptor (PR), and human epidermal growth factor receptor 2 (HER2). TNBC accounts for 15% to 20% of all breast cancer pathology types, with low-grade particular variants like secretory carcinoma and adenoid cystic carcinoma having a good prognosis. On the other hand, high-grade malignancies such spindle cell metaplastic carcinoma and basaloid carcinoma have a poor prognosis.

Triple-negative breast cancer is more common in premenopausal women, and it is also a specific molecular subtype of breast cancer in clinical practice [6]. Breast cancer that is triple-negative progresses quickly and is invasive. The cancerous breast cells are loosely connected, and cancer cells are efficiently distributed throughout the body along with the lymphatic system and blood circulation, resulting in cancer metastasis, which not only increases the difficulty of treatment but also has a particular impact on the health of patients [7–9]. Furthermore, modern women are under more physical and emotional stress, which has resulted in an increase in the prevalence of breast cancer, particularly triple-negative breast cancer. All of the receptors for human epidermal symptom factor 2, progesterone receptors, and estrogen receptors are negative. This is the term for triple-negative breast cancer [10–12]. Furthermore, triple-negative breast cancer is aggressive, with a high risk of recurrence, distant metastasis, and visceral and bone metastases. Breast cancer that is triple-negative has a poorer prognosis than other types of breast cancer [13–15]. Because there is no known specific treatment for TNBC, it is currently usually treated with chemotherapy. Once metastasis and dissemination have occurred, TNBC patients have a 5-year survival rate of less than 30%. As a result, for triple-negative breast cancer patients, early detection is critical [16, 17].

In clinical practice, there are several diagnostic programs for triple-negative breast cancer, and X-ray irradiation exposes the body to a significant quantity of radiation. Magnetic resonance imaging (MRI) is a noninvasive operation. 3.0 T MRI can determine the morphological information of breast cancer and evaluate the tumor function and the surrounding blood vessels of the tumor [18–20]. It has a high application value for triple-negative breast cancer. This method has a high application value [21–24]. The molecular typing of breast cancer is generally diagnosed by an immunohistochemical examination of patients, which is complicated and invasive. Therefore, some researchers try to predict the molecular type of breast cancer through patient images. The imaging techniques mainly include mammography, breast ultrasound, positron emission tomography, and dynamic enhanced magnetic resonance. These techniques generally use artificial extraction of features, and these are subjective. It is difficult to objectively reflect the essential characteristics of breast cancer [25, 26].

Today, deep learning methods are applied to many pattern recognition tasks with good results, in which convolutional neural network algorithms can automatically learn image features [27]. Men et al. [28] presented DD-ResNet, an end-to-end deep learning model that allows for quick training and testing. The authors then evaluated an extensive dataset of 800 patients receiving breast-conserving therapy. The authors found that the model can achieve good segmentation results. By creating two fully convolutional neural networks (CNNs) based on SegNet and U-Net tumor segmentation, two deep learning techniques were proposed by El Adoui et al. [29] to automate breast imaging in dynamic contrast-enhanced magnetic resonance imaging (DCE-MRI). For a convolutional neural network (R-CNN) network, Lei et al. [30] built a backbone network, a region proposal network, a region convolutional neural network head, a mask head, and a scoring head. The network properly segments breast cancers. Singh et al. [31] proposed a breast tumor segmentation method based on a contextual information-aware conditional generative adversarial learning framework. The approach extends a deep adversarial learning framework by collecting texture information and contextual dependencies in tumor photographs to achieve successful breast segmentation.

This study presents a fully automated segmentation method based on a convolutional neural network algorithm and SVM. The framework is split into two sections. In the initial stage, the CNN is taught mapping from image space to tumor label space. To accomplish accurate segmentation in the testing phase, the CNN's predicted label output is used and combined with the test grayscale picture in an SVM classifier. After the SVM classifier, a more accurate binary segmentation image can be obtained. In recent years, the algorithm combining CNN and SVM has been proposed in much literature. The algorithm described in this work is primarily distinct from the CNN research approach when compared to other integrated algorithms. The N4ITK method, with ReLU as the activation function, negative log-likelihood loss function as the loss function, stochastic gradient descent as the optimization strategy, and so on, is employed as a preprocessing technique in this study. Furthermore, to improve the quality of the features retrieved from CNN, they are sent to the SVM classifier. This paper also includes a stage of intermediate processing that improves segmentation.

## 2. Materials and Methods

### 2.1. Construction of the Dataset

#### 2.1.1. Data Acquisition

We collected breast MRI data from 272 patients from the Second Affiliated Hospital of Fujian Medical University. There were 165 cases of other molecularly pressed breast cancer and 107 triple-negative breast cancer cases. The inclusion criteria were as follows: (1) breast MRI examination was performed before surgery. (2) The postoperative pathology report accurately indicated the molecular subtype of breast cancer. MRI were collected utilizing a specialized phased array 8-channel breast coil on a 3.0 T MRI scanner (PHILIPS, Ingenia 3.0 T) with patients in the prone position. The identical imaging strategy was used on all of the patients. The breast DCE-MRI protocol included an axial T2-weighted Fast Spin Echo (T2-FSE) sequence (Repetition Time/Echo Time (TR/TE) = 3600/100 ms, flip angle = 90°, matrix size = 512 × 512, and slice thickness = 4.0 mm) and an axial Short Tau Inversion Recovery (STIR) sequence (TR/TE = 3900/90 ms, flip angle = 90°, and matrix size = 512 × 512). The DWI methodology included a DWI sequence (TR/TE = 6000 ms/90 ms, flip angle = 90°, matrix size = 256 × 256, slice thickness = 4.0 mm, and *b* values of 0 and 850 s/mm^2^) collected before the contrast material was injected.  Figure 1 depicts a portion of the scanned picture data.

#### 2.1.2. Data Annotation

Two senior medical radiologists engaged in breast imaging diagnosis manually delineated the tumor images we collected. The molecular subtype labeling was the gold standard based on the pathology report. In addition, corresponding contour labels are also made according to the boundaries of the tumor labels. The boundary of the contour label is represented by 1, and the area outside the boundary is represented by 0. Because Bayesian field distortion alters the MRI picture, the gray value of the same spot in the image will be unequal. We utilized the N4ITK approach to solve this issue.

At the same time, we also performed block extraction on the data. In this paper, each pixel in the image is taken as the center to extract a two-dimensional data block as training data. The retrieved data block is separated into positive and negative samples based on the label of the center pixel, according to the gold standard for tumor segmentation. Tumor areas correlate with positive samples. The nontumor region, i.e., the normal tissue structure of the chest, corresponds to the negative samples. Because the lesion area is significantly less than the normal tissue region in practice, the number of negative samples far outnumbers the number of positive samples. A random downsampling strategy is used to balance the quantity of positive and negative data submitted to the training model. Make the block size 17 by 17 inches.

### 2.2. Convolutional Neural Network Model Implementation

A convolutional neural network [32] is essentially a multilayer perceptron with additional layers. It is a multilayer neural network design. There are three levels to it: an input layer, a hidden layer, and an output layer. In the hidden layer, there might be several levels. Each layer is made up of a number of two-dimensional planes, each containing a number of neurons. A feature extraction layer and a subsampling layer are stacked in the concealed layer.  Figure 2 depicts the structure of a convolutional neural network. Here are some of CNN's most important features.

The activation function uses a linear correction unit (ReLU), which is defined as

(1) $$\begin{array}{c} f\left(x\right)=\max\left(0,x\right). \end{array}$$

It is found that the algorithm using ReLU can achieve better results and faster training speed than the traditional sigmoid or hyperbolic tangent function [33]. A softmax classifier was used for 2-class classification when using CNN alone for segmentation.

This paper uses max pooling [34], which computes the maximum value of a particular feature in an image region. This solves the problem that after the features are obtained by convolution if all the extracted features are used for training, the calculation will increase, and it is easy to overfit.

Regularization is used in this research to reduce overfitting. When utilizing CNN alone for segmentation, dropout technology is used in the FC layer to clear the output value in the hidden layer node with a probability of 0.2 to reduce the dependency between the hidden layer nodes. This is a good approach to prevent overfitting.

The loss function, in its most basic form, is the function that is used to calculate the training model's error. In general, it is intended that this function may be reduced to the bare minimum. The negative log-likelihood loss function is used in this study, and it is defined as

(2) $$\begin{array}{c} \text{NLL}\left(\theta ,D\right)=-\overset{\left|D\right|}{\underset{i=0}{\sum }}\log P\left(Y=y^{\left(i\right)}\left|x^{\left(i\right)},\theta \right.\right). \end{array}$$

### 2.3. SVM Principle

Based on statistical learning theory, VC dimension theory, and structural risk reduction criterion, support vector machine is a supervised learning strategy that attempts the best balance between model complexity and learning capacity. It can gain lower real risk and has a great generalization capacity [35]. When using SVM to solve nonlinear classification problems, the inner product kernel function replaces the nonlinear mapping to the high-dimensional space rather than the dimension of the sample space, avoiding the problems that traditional learning classifiers can encounter when dealing with nonlinear high-dimensional problems. It is difficult to keep track of the digits. The support vector machine's goal is to discover the optimal hyperplane for feature space division, and it works on the maximization of the classification interval concept. The minimization function for determining the best hyperplane margin and associated restrictions is defined by equations (3) and (4) and (3)–(5).

(3) $$\begin{array}{c} \underset{w,b}{\min}\frac{1}{2}{\left\|\overset{⟶}{w}\right\|}^{2}, \end{array}$$

subject to the constraints

(4) $$\begin{array}{c} y_{i}\left(\overset{⟶}{w}∙\overset{⟶}{x_{i}}+b\right), \end{array}$$

where *w* is the normal, *b* is the threshold, and *x*_*i*_ is each sample instance.

The optimal classification surface or optimal classification line should separate the two types of samples without error and maximize the classification interval of the two types, which is the essential requirement of the structural risk minimization criterion. The purpose of separating the two types of samples without errors is to minimize the empirical risk; maximizing the classification interval of the two types ensures that the classifier has the smallest VC dimension and thus obtains the smallest confidence range, so that the classifier has the least real risk. The optimal classification surface of the SVM method is unique.

The support vector machine in this work uses the Gaussian radial basis kernel function, which is defined as

(5) $$\begin{array}{c} K\left(x,x_{i}\right)=\exp\left(-\frac{{\left\|x-x_{i}\right\|}^{2}}{\sigma^{2}}\right). \end{array}$$

At this time, the support vector machine is a radial basis function classifier, which is different from the traditional radial basis function technique, and its weights are produced automatically.

### 2.4. Breast Tumor Segmentation Based on the CNN-SVM Combined Model

This study proposes a brain tumor segmentation approach based on a convolutional neural network and SVM. Preprocessing, feature extraction, CNN and SVM training, and testing and providing final segmentation results are the major steps of the proposed architecture, as shown in Figure 3.

Convolutional neural networks and support vector machines are trained separately in the first stage to learn the mapping from the grayscale picture domain to the tumor label domain. During the testing phase, the SVM classifier receives the labeled output of the convolutional neural network as well as the test grayscale picture for accurate segmentation. A simple intermediate processing step is introduced to create relevant features for CNN training, as illustrated in Figure 4. To represent each pixel, we employ first-order characteristics (grayscale, mean, and median). A CNN is taught utilizing these properties during the training phase to learn a nonlinear mapping between input information and labels. The SVM classifier is trained independently during the testing phase, using the CNN label map and the same features as before.

### 2.5. Model Design Details

Softmax is a multiclass classifier used here for 2-class classification whose output is a conditional probability value between 0 and 1. The convolutional neural network structure proposed in this paper consists of a convolutional layer, a pooling layer, a fully connected layer, and a softmax classification layer, where softmax is a multiclass classifier used here for 2-class classification whose output is a conditional probability value between 0 and 1.

ReLU is used in the network's transfer function. The stochastic gradient descent technique is used to get the network parameters and model by minimizing the loss function. The network's input image data block is 17 × 17 bytes long. After the first convolution layer C1, 32 filter templates of size 5 × 5 are used for convolution to obtain 32 feature maps of size 13 × 13, and then, the maximum pooling is performed. With sampling layer S2, use 2 × 2 template nonoverlapping pooling to obtain 32 feature maps of size 66, and then, through convolution layer C3, use 64 filter templates of size 3 × 3 convolutions to obtain 64 sizes. It starts with a 2 × 2 feature map, then downsamples S4 using the maximum pooling of the 2 × 2 templates, then converts each feature map into a single neuron node using 128 2 × 2 filter template convolutions, and lastly links all of them together. At the connection layer F6, some tumor edge and texture features will be acquired from the network, and the low-level features will be converted into high-level features after multilayer learning. Finally, intermediate preprocessing is performed to give the SVM classifier the obtained high-level features. Each pixel in the image is sorted into two groups based on the likelihood value of the category to get the probability value of tumor or normal chest tissue. Size classification is utilized to create a segmented binary image of the tumor.

With the increase in the window size, the correct rate of SVM classification samples will decrease, and the effect is better when the window size is small. At the same window scale, the segmentation results of SVMs with different kernel functions are not much different.

The SVM technique using polynomial kernels, on the other hand, yields slightly poorer results than the linear kernel and radial basis kernel SVM methods. In addition, we set *C* = 1, 10, 100, 1000, and 10000 and *σ*^2^ = 0.01, 0.125, 0.5, 1.5, and 1.0, respectively, for sample training and found through experimental data that when *C* is set between 100 and 1000, when *σ*^2^ is set between 0.01 and 0.125, the cross-validation accuracy is the highest. As a result, when utilizing the radial basis kernel function to offer the best segmentation results, the penalty factors *C* and 2 should not be too little or too large. As a consequence, we chose *C* = 1000, *σ*^2^ = 0.01, 5 × 5 as the window size, and 2000 as the training sample count.

## 3. Results

### 3.1. Evaluation Metrics

Dice Similarity Coefficient (DSC) is an index that measures the rate at which manual and automatic segmentation is repeated. It is defined as follows:

(6) $$\begin{array}{c} \text{DSC}=\frac{2\text{TP}}{\text{FP}+2\text{TP}+\text{FN}}. \end{array}$$

The number of tumor sites identified as true positive, false positive, and false negative, respectively, is denoted as TP, FP, and FN.

Positive predictive value refers to the ratio of correctly segmented tumor points to the segmentation result of tumor points (PPV), which is defined as

(7) $$\begin{array}{c} \text{PPV}=\frac{\text{TP}}{\text{TP}+\text{FP}}. \end{array}$$

The percentage of successfully segmented tumor points to the real value of tumor points is known as sensitivity, and it is defined as

(8) $$\begin{array}{c} \text{Sensitivity}=\frac{\text{TP}}{\text{TP}+\text{FN}}. \end{array}$$

### 3.2. Segmentation Results of the CNN-SVM Model

We train and segment the gathered breast tumor photos and present the experimental findings to demonstrate the CNN-SVM model's segmentation effect. The segmentation impact is clearly visible in the ensuing graph, demonstrating the efficacy of our strategy. The segmentation results of image slices of triple-negative breast cancer samples are shown in Figure 5.

At the same time, to verify our method's effectiveness again, we randomly selected several samples from the scanned images of other types of breast cancer for testing.  Figure 6 shows the segmentation results of image slices of other types of breast cancer samples.

As can be seen in the diagram, our network is capable of successfully segmenting breast cancers. As a result, our network is extremely successful in segmenting breast cancers.

### 3.3. Comparison with Existing Methods

To demonstrate the usefulness of our suggested approach, we compare it to methods offered by other researchers, and the results of the comparison are presented in Table 1. To segment breast cancers, Byra et al. [36] designed a Selective Kernel (SK) U-Net convolutional neural network. Rouhi et al. [37] used convolutional neural networks for breast tumor segmentation. Haq et al. [38] proposed an automatic breast tumor segmentation method using conditional GAN (cGAN). Table 1 shows that the CNN-SVM combination model developed in this study outperforms other approaches in terms of DSC, PPV, and sensitivity, demonstrating the practicality of our strategy.

## 4. Discussion

Breast cancer is increasing at a rate of 3% to 4% every year, and it has become the first cancer-related death among women. Most of them go to the hospital for treatment only after symptoms, and they have the worst understanding of the census. The etiological factors of this disease include oral contraceptives, a high-fat diet, heavy drinking, obesity, long-term smoking, and unstable ovarian function, which seriously affect patients' quality of life and increase the economic burden on patients. As a result, it is vital to diagnose and treat people with breast cancer or suspected breast tumors as soon as possible. In recent years, MR is often used to diagnose breast cancer. Most studies have shown that 3D imaging of MRI has the advantages of multiparameter and multiplanar imaging and has a higher soft tissue resolution. Compared with mammography, MRI can more accurately display the type of lesions and tumor staging. At the same time, MRI dynamic contrast-enhanced scanning has high diagnostic sensitivity and accuracy and can well present high breast lesions, deep lesions, and multifocal lesions. In addition, this inspection method can show the morphological changes of the mass and reflect the microvascular perfusion and angiogenesis of the mass through dynamic enhanced scanning to effectively evaluate the malignancy of the mass and facilitate grading diagnosis.

Based on a convolutional neural network method and SVM, we present a hybrid network for complete automatic segmentation. The network is made up of two phases that are linked together. The CNN is trained initially to learn the mapping from image space to tumor label space. The anticipated label output from the CNN is then added to an SVM classifier together with the test grayscale picture to obtain correct segmentation. A more accurate binary segmentation picture can be obtained after the SVM classifier.

Similar to other researchers, our method also suffers from certain limitations. First, the accuracy of data annotation needs to be improved, and the size of the dataset needs to be expanded. Existing medical imaging data is primarily labeled by hand, which necessitates a significant amount of people and material resources. The accuracy of labeling is closely related to the level of doctors, so the quality of datasets is uneven. In addition, the private nature of medical images also makes it difficult to obtain data. Doctors at the hospital use regular sketching software to annotate the obtained annotation dataset. The annotation quality must be enhanced, and the quantity of MRI pictures must be increased. Secondly, the network performance also needs to be improved, reducing the number of parameters and speeding up the training speed. The segmented breast tumor may be reconstructed into a three-dimensional model [39] for better visualization. In addition, one may use extreme learning techniques [40, 41] for the segmentation to compare against our proposed method in future implementation.

## 5. Conclusion

For MRI breast tumor segmentation, this research presents a CNN-SVM network. The label output of a learnt convolutional neural network is guided into a support vector machine in this technique. The convolutional neural network and the support vector are trained separately in the training phase to learn the mapping from the grayscale picture domain to the tumor label domain. The SVM classifier receives the labeled output of the convolutional neural network and the grayscale picture of the test for correct segmentation in the testing stage. In future study, we will look at convolutional neural networks paired with additional robust classifiers. When compared to previous studies' segmentation frameworks, the DSC, PPV, and sensitivity of our CNN-SVM combined network are 0.93, 0.95, and 0.92, respectively, indicating that it has higher segmentation performance and can accurately segment breast cancers. The diagnosis of breast cancer by medical elastography can be further enhanced with the possibility of implementing optical flow motion analysis on the MRI scans [42, 43] and identifying the regions of abnormal stiffness.

## Figures and Tables

**Figure 1:** Partially scanned image based on the (a) T2 scan sequence and (b) DWI scan sequence.

**Figure 2:** CNN network structure diagram.

**Figure 3:** Algorithm framework of breast tumor segmentation based on the combination of CNN and SVM.

**Figure 4:** Intermediate processing steps.

**Figure 5:** Image slice segmentation results of triple-negative breast cancer samples based on (a) raw MRI scan image, (b) segmentation results of CNN-SVM, and (c) real image segmentation result.

**Figure 6:** Image slice segmentation results of other types of breast cancer samples based on (a) raw MRI scan image, (b) segmentation results of CNN-SVM, and (c) real image segmentation results.

**Table 1:** Comparison of different algorithms.

Method	Literature	DSC	PPV	Sensitivity
U-net	Byra et al. [36]	0.88	0.89	0.90
CNN	Rouhi et al. [37]	0.90	0.92	0.89
BTS-GAN	Haq et al. [38]	0.92	0.93	0.91
CNN+SVM	Our method	0.93	0.95	0.92

## Data Availability

Data are available on request from the authors due to privacy/ethical restrictions.
